The article "The Use of Coercive Interventions in Mental Health Care in Germany and the Netherlands. A Comparison of the Developments in Two Neighboring Countries" was published in 2014. Journal: Front Public Health.

# The Use of Coercive Interventions in Mental Health Care in Germany and the Netherlands. A Comparison of the Developments in Two Neighboring Countries

**DOI:** 10.3389/fpubh.2014.00141

**Published:** 2014-09-24

**Authors:** Tilman Steinert, Eric O. Noorthoorn, Cornelis L. Mulder

**Affiliations:** ^1^Centre for Psychiatry Suedwuerttemberg, Ulm University, Ulm, Germany; ^2^Dutch Case Register on Coercive Measures, Expertise Centre for Aggression Management, Den Dolder, Netherlands; ^3^Epidemiological and Social Psychiatric Research Institute, Erasmus MC, Rotterdam, Netherlands

**Keywords:** coercion, seclusion, restraint, involuntary commitment, enforced medication, community treatment order, involuntary outpatient treatment, guideline

## Abstract

In this review, we compare the use of coercion in mental health care in Germany and in the Netherlands. Legal frameworks and published data on involuntary commitment, involuntary medication, seclusion, and restraint are highlighted as well as the role of guidelines, training, and attitudes held by psychiatrists and the public. Legal procedures regulating involuntary admission and commitment are rather similar, and so is the percentage of involuntary admissions and the rate per 100,000 inhabitants. However, opposing trends can be observed in the use of coercive interventions during treatment, which in both countries are considered as a last resort after all other alternative approaches have failed. In the Netherlands, for a long time seclusion has been considered as preferred intervention while the use of medication by force was widely disapproved as being unnecessarily invasive. However, after increasing evidence showed that number and duration of seclusions as well as the number of aggressive incidents per admission were considerably higher than in other European countries, attitudes changed within recent years. A national program with spending of 15 million € was launched to reduce the use of seclusion, while the use of medication was facilitated. A legislation is scheduled, which will allow also outpatient coercive treatment. In Germany, the latter was never legalized. While coercive treatment in Germany was rather common for involuntarily committed patients and mechanical restraint was preferred to seclusion in most hospital as a containment measure, the decisions of the Constitutional Court in 2011 had a high impact on legislation, attitudes, and clinical practice. Though since 2013 coercive medication is approvable again under strict conditions, it is now widely perceived as very invasive and last resort. There is evidence that this change of attitudes lead to a considerable increase of the use of seclusion and restraint for some patients.

## Introduction

Mental disorders are by definition mental and behavioral disorders. Severe deviations of behavior such as violent, suicidal, and many other features of bizarre and inappropriate behavior belong to typical symptoms of mental disorders. Up to nowadays, besides of psychotherapeutic and pharmacological interventions, the use of coercion is sometimes considered as inevitable in managing dangerous and severely disturbing behavior. The issue of coercion with its many facets is the oldest problem of psychiatric institutions. The history of psychiatry is essentially characterized by attempts to abolish coercion and by failing of such attempts, up to episodes of excessive violence against mentally ill people such as during the Nazi regime in Germany (1). Not accidentally, the beginning of psychiatry as a medical discipline has been dated in textbooks of history to the liberation of the inmates of the French hospitals Bicêtre and Salpétrière from their chains by Philippe Pinel in Paris in 1793. In the second half of the nineteenth century, the no-restraint movement, initiated by Connolly and Hill in England, aimed for the total abolition of compulsory measures in the treatment of mentally ill people (2). This aim of no-restraint led to controversy and ongoing discussions in several European countries at the time. Effectively, the complete abolition of coercive interventions has never been convincingly reported in any country or period. However, the discussion is still alive nowadays and has become increasingly important due to several reasons. The public and the mass media are concerned simultaneously (and contradicting) about patients’ rights and respect for their dignity on the one hand and dangers imposed to the public by people with severe mental illness who account for a non-neglectable proportion of violent deaths (3) on the other hand. People with severe mental illness have been identified as a particularly vulnerable population for the violation of human rights by the European Committee for the Prevention of Torture and inhuman or degrading Treatment (CPT). More recently, the UN-Convention on the Rights of Persons with Disabilities, which has been acknowledged by the European Union in 2008, emphasized the rights of such vulnerable populations. In 2013, a report of the special rapporteur on torture and other cruel, inhuman or degrading treatment or punishment to the United Nations’ general assembly, claimed to definitely ban restraint, seclusion, and involuntary treatment (4).

Thus maybe the most fundamental ethical conflict in clinical psychiatry exists between the ethical principles of respect for the patient’s autonomy and dignity and the duty to avoid harm for the patient and others. The undesirable result of this conflict sometimes is the use of coercion, which can occur in many different aspects of psychiatric treatment – coercive admission to psychiatric hospitals, safety measures within psychiatric institutions, coercive treatment inside and outside psychiatric hospitals, referral to forensic psychiatric units, and more. All of these measures are increasingly under regulation of laws, court decisions, guidelines, and ethical considerations, and have repeatedly been a subject of concern in the public and in the media in many developed countries. Moreover, within recent years, digital data processing from electronic charts has provided the possibility to discuss the issue of coercion in psychiatry not only based on qualitative arguments but also based on data covering the practice of mental health care.

Germany and the Netherlands are neighboring countries with a comparable social structure, comparable social standards, and roughly similar politics, both being confronted with similar challenges to find appropriate, human, and safe solutions for the use of coercion in mental health care. The challenge is to balance requirements and expectations of patients, relatives, hospital staff, the justice systems, policy makers, and society as a whole. In this article, we will elucidate the current practice in both countries, the differences and how they emerged and interactions with learning from each other’s practice.

## Method

According to the complexity of the issue, this is a review based essentially on personal knowledge of the authors who had a kind of central role in collecting and interpreting data and phrasing clinical recommendations in the respective country. The literature review covers the relevant publications of the last decade. It is amended by knowledge of relevant court decisions, policies, clinical guidelines, legislation changes, initiatives, and current, still unpublished developments. We selected 10 topics related to the use of coercion, which taken together to cover the relevant aspects sufficiently.

## Legislation

### Germany

Coercive interventions in psychiatry are regulated in the law of guardianship (Betreuungsrecht), as a federal law valid everywhere in the country, and in the public laws (comparable to Mental Health Act in other countries) with slightly different regulations in the 16 German federal states (Bundesländer) (PsychKG, UBG) (5). It had been expected since about a decade that it would be necessary to consider involuntary admission and involuntary treatment separately in law texts as it is realized in some European countries and in the United States already since 1980 (6, 7). This happened with two decisions of 2011 of the Constitutional Court (Bundesverfassungsgericht) on involuntary medication in forensic psychiatry, which had a huge impact on clinical practice. In two cases, the Constitutional Court decided that the existing laws regulating involuntary medication were unconstitutional and thus no more valid. The Constitutional Court claimed that law texts should clarify that involuntary medication should be applied only for people without capacity to consent, only as a last measure if all other approaches have failed, only under strict circumstances and only after a separate court decision, taking into account the opinion of an independent expert. Though this decision primarily related to forensic psychiatry, other Supreme Courts (Bundesgerichtshof) adopted this view and extended it to all kinds of involuntary treatment also for civil patients. Consequently, involuntary medication was no more possible except for acute emergencies until in 2013 new legislations fulfilling the requirements of the Constitutional Court were adopted. This referred to guardianship law and public law as well. Adoption of legislation is still under way in several German federal states. The German Psychiatric Association (DGPPN) explicitly appreciated the Constitutional Court’s decision and declared that it was comprehensively in line with the conception of medical ethics (8). Another new legislation relates to the use of technical coercive measures, which until recently have been only poorly regulated by law. In 2012, the law for the ban of video surveillance was adopted in Nordrhine-Westphalia, prescribing 1:1 surveillance during mechanical restraint or seclusion. Other German federal states are preparing similar laws.

### The Netherlands

Currently, the Law for special admissions in psychiatric hospitals Bijzondere Opnemingen Psychiatrische Ziekenhuizen (BOPZ) primarily regulates admission and allows coercive interventions to some extent under strict conditions. The law contains two different sections describing the procedures of involuntary admission. The first relates to short-term involuntary admission because of immediate danger for the patient himself or others and has to be initiated by the mayor, accompanied by a written certificate of a physician. The other procedure is mandated by a judge and concerns long-term admissions aiming at treatment of patients who suffer from a severe psychiatric disorder leading to danger for others or self, including severe self-neglect or social breakdown. After involuntary admission, community treatment orders can be used.

This law regulates explicitly, which measures are possible in case of emergency. Seclusion, mechanical restraint, and enforced medication may be applied for no more than 7 days. Actions taken are communicated to the Dutch health inspectorate. If coercive measures are required for more than 7 days, a treatment plan has to be established and has to be approved by a psychiatrist not involved in treatment. The patient can take legal action also against the independent psychiatrist’s second opinion. In practice, procedures associated with coercive treatment can be complex and time consuming and may delay remission if a patient is reluctant to accept treatment. This law is effective since 1994.

Psychiatrists have to document, which measures were taken and are obliged to use the least restrictive method. According to a governmental order of 2012, documenting all coercive measures at an accuracy of 15 min is mandatory, allowing for a nation-wide registration of coercive measures and careful monitoring at ward, hospital, and national level (9). In 2008, regulations with respect to community treatment orders were extended.

## Involuntary Outpatient Treatment

### Germany

Involuntary outpatient treatment has never been legalized in Germany. Only in 2003, the Federal Council (Bundesrat) passed a draught legislation, which provided an amendment to the guardianship law, allowing delivery of outpatients to treatment by force. However, after some intense political debates and strong objections by patients’ organizations, the Federal Parliament (Bundestag) rejected the draught law in 2004. Community treatment orders are possible only for former forensic patients in specialized outpatient services for these patients.

### The Netherlands

Under the current Dutch law involuntary outpatient treatment, i.e., administering drugs by direct coercion, is not legal. However, it is possible to mandate community treatment orders. If the patient does not comply with the conditions of the outpatient treatment order, involuntary admission can be immediately put into effect. Besides of taking prescribed drugs, the patient can be obliged to visit outpatient services at regular intervals, and keeping to appointments. Violation of these obligations can lead to an immediate search warrant by the local authorities followed by an involuntary admission. In the near future, Dutch law will allow involuntary outpatient treatment irrespective of admission under two separate laws for patients with a psychiatric illness and patients with a mental handicap or a severe old age impairment.

## Coercive Hospital Admission and Involuntary Commitment

### Germany

Hospital admission under coercion is possible under different pathways: by a court decision, by decision of the police in some German federal states and, more informally, but not unfrequently, by psychological pressure of doctors and relatives. Thus no reliable data on the frequency is available. Some earlier publications probably merged involuntary admission with involuntary commitment (10). Involuntary commitment is clearly defined by a court decision. There are three different types of relevant court decisions: Commitment to forensic psychiatry due to an offense in state of decreased or annihilated criminal responsibility, civil commitment under guardianship law due to danger to self and civil commitment under public law (Mental Health Act) due to acute danger to self or others.

The number of patients detained in forensic psychiatry in Germany increased about 2.5-fold from about 4,000 in 1993 to about 10,000 in 2009 (11), similarly to many other developed countries (12). However, the development was considerably different among the German federal states (11). In-depth analyses showed that the bulge was mostly due to an increase of referrals of psychotic patients with non-letal violent crimes (13).

In a study comparing involuntary placements of mentally ill people across EU member states, the number of civilly committed patients was determined as 163,000 in the year of 2000, yielding a rate of 175 per 100,000 population and a quota of 17.7% of all psychiatric admissions. The rate was one of the highest in a range between Portugal (6/100,000) and Finland (218/100,000), and even so the quota, ranging from 3.2% (Portugal) to 30% (Sweden) (6). However, the most recent very comprehensive data collection indicated considerably lower figures (rate 131/100,000, quota 10% of all admissions) for the same year. The most topical available data from the year 2009 (14) is displayed in Table 1.

**Table 1:** **Involuntary commitment in Germany 2009 [according to Ref. (14)]**.

	Prevalence in 2009	Change since 1994 (%)
Total rate per 100,000	171.9	+42
Rate by guardianship law	84.9	+160
Rate by mental health act	87	+17
Total quota of admissions	10.9%	−10
Quota of admissions committed according to guardianship law	4.72%	+4
Quota of admissions committed according to mental health act	6.21%	−14

Again, there are considerable and not convincingly explained differences between the 16 German federal states (14), rates and quotas being lower in the 5 new (former German Democratic Republic) states. The data displayed in Table 1 indicate that the rates of involuntary commitment have been considerably (and continuously) rising within the 15 years observed, while the quota of all psychiatric admissions has even decreased. This is due to the fact that the number of psychiatric admissions has also been continuously increasing during this period, even slightly more than the number of involuntary commitments, so that the percentage of involuntary patients among psychiatric hospital patients is even declining in spite of an increasing percentage of the population being subjected to involuntary commitment (14).

### The Netherlands

As stated above, in the Netherlands, hospital admission is regulated in a special law regulating involuntary admissions in psychiatric hospitals (Law BOPZ). As in Germany, admissions to forensic settings can be mandated after a criminal offense, by the “law regulating principles of care for people under governmental mandate” (beginselenwet verpleging ter beschikking gestelden). Table 2 depicts the Dutch developments for short-term and long-term involuntary commitment according to this law, separated into rates and quotas according to the data from Germany, indicating a considerable increase of long-term involuntary admissions within the past 10 years.

**Table 2:** **Involuntary commitment in the Netherlands 2009 (15)**.

	Prevalence in 2013	Change since 2002 (%)
Total rate per 100,000	136	+65
Rate by short-term involuntary admission	47	+8
Rate by long-term involuntary admission	89	+86
Total quota of admissions	10.8%	+23
Quota of admissions by short-term detention	3.8%	+8
Quota of admissions by long-term involuntary admission	7%	+128

## Involuntary Medication and other Involuntary Treatment

### Germany

As mentioned above, in 2011 the Constitutional Court (Bundesverfassungsgericht) decided that the current laws are unconstitutional. Data how frequently involuntary medication really happened until then is not available, amongst others due to the lack of clear definitions. From then on, involuntary medication was only possible in cases of acute emergency until the novel law formulation was adopted by the parliament (Bundestag) in the beginning of 2013. Thus currently involuntary medication is possible after a distinct court decision and an expert opinion by a doctor not involved into treatment. Data on how frequent such kind of involuntary medication and also medication in emergencies happens is not yet available. It is known from anecdotal evidence that sometimes procedures are very long and cumbersome resulting in periods of weeks or even months with patients being committed without receiving treatment. The latter is a point of concern for psychiatrists with respect to ethical considerations and ward atmosphere (8). Involuntary medication has been an issue of a strong and controversial debate after 2011 in the public and among professionals as well, fueled by very pointed statements of anti-psychiatric patient’s organizations and an appeal to the German parliament by the German Institute of Human Rights not to pass any legislation allowing involuntary medication in psychiatry (16). Fears expressed by psychiatrists that a restriction of the use of medication would lead to an increase of mechanical containment measures such as seclusion and restraint and to an increase of violent incidents recently are supported by evidence from observational studies (17).

### The Netherlands

According to Dutch law, a psychiatrist has to apply the least invasive approach in dealing with aggression or other behavior, which is dangerous for the patient himself or others. The patient’s mental capacity and ability to balance decisions determine the extent to which psychiatrists are allowed to impose treatment against a patient’s will. In the Netherlands, involuntary medication was traditionally viewed as a more invasive approach than the use of seclusion, so that the frequency of its use was only a fourth of the use of seclusion after implementation of the law for special admissions (18, 19). With the change in legislation to come in mind, but also being aware of more data on the practice in other countries, Dutch hospitals’ policy makers as well as the Dutch mental health inspectorate in recent years have been changing their attitude from a clear preference of seclusion to a more differentiated choice of measures, based on international literature (20). However, the Dutch health inspectorate as well as the government both have issued reports as well as policies, cautioning hospitals not to replace one coercive measure by another. In a letter to hospital directors, the minister of health warned that sanctions to the hospitals by the Health inspectorate might follow if enforced medication should replace seclusion as a measure to deal with aggression. This primarily political claim is difficult to implement against the background of available evidence, which suggests that use of mechanical measures such as seclusion is inversely associated with the use of medication (21–23). Despite these strong political recommendations, according to the law decisions lie with the treating psychiatrist and the medical director. Their policy in case of involuntary treatment is reviewed by the mental health inspectorate. If they carefully document their choices, the law allows them to do so, even against the general feeling in the Dutch political context.

## Seclusion

### Germany

There is some data available on the use of freedom-restrictive coercive measures in psychiatric hospitals, but only very little data indicating whether the measure used is seclusion or mechanical restraint. Anecdotal evidence indicates that seclusion is considered as the measure of choice in child- and adolescent psychiatry and in forensic psychiatry, while in adult general psychiatry many hospitals prefer to use mechanical restraint and a considerable number does not provide seclusion rooms. A survey of the use of coercive interventions in psychiatric hospitals in Germany in 2012 revealed that 51% of the responding hospitals used seclusion, 53% with continuous observation, and 16% without continuous observation. However, these figures have to be interpreted with caution since the response rate of this survey was only 20% (24). Data on the frequency of such freedom-restrictive coercive measures will be reported in the next section.

### The Netherlands

Traditionally, and especially after a change in the Dutch mental health act, seclusion was the coercive measure of first choice in the Netherlands (9, 25). Between 1994 and 2006, data collected on the number and the duration of seclusions showed high figures in comparison to other European countries. In 2004, a study performed in 12 hospitals showed that 60% of the measures taken were not reported to the Health inspectorate. Also, approximately 27% of patients on admission wards were subjected to seclusion and the duration was estimated 250 h per patient (26). This finding, presented in 2004, lead to a national uproar. In 2005, a program of 15 million € was launched by the Dutch Government to stimulate hospitals in efforts to reduce seclusion and restraint by 10% per year. Since then, a trend analysis showed a clear reduction in the use of seclusion, though the objective of a 10% reduction per year was not achieved (19).

After 2007, an increasing number of hospitals have registered their data in a daily database on the use of coercive measures; this database is now available on a national level. The database was designed similarly to the database developed by the German working group for prevention of violence and coercion in psychiatry (27). In the database, the number and duration of measures of seclusion and restraint is related to admission data with respect to age, marital and ethnic status, diagnosis, and admission hours. Findings show a steady decrease of exposure to coercive measures, from 13.2% of admitted patients in 2008 to 9% in 2012. Seclusion dropped from 11.2 to 6.5%. In the same time, the sample increased from a selected population of eight hospitals in 2008, over a representative sample in 2010, to a near to nation-wide coverage in 2012 (Table 3). While the first 14 hospitals in 2008 and 2009 covered about 14,900 patients and 23,000 admissions (28), the findings gathered in 2012 covered 130,000 admissions and over 59,000 patients.

**Table 3:** **Nation-wide registration of coercive measures: seclusion figures 2008–2012**.

Year	Hospitals	Wards (*N*)	Seclusions	Exposure (%)	Exposed patients (*N*)	Hours		Decrease hours seclusion/admission hours between years^a^ (%)
						Mean	Median	
2008	8	68	3685	11.2	1671	128	92	−45

2009	14	198	5525	10.8	2322	71	43	

2010	18	227	4750	10.2	2722	70	38	−17

2011	21	375	7476	8.5	3743	62	35	−17

2012	53	506	9469	6.5	7198	58	17	−13.5

*^a^Comparison 2008–2012 in sample of 2008, 2009–2012 in sample of 2009, 2010–2012 in sample of 2010, and 2011–2012 in sample of 2011*.

## Mechanical Restraint

### Germany

Mechanical restraint has been considered as the measure of choice in the management of violent behavior in general adult psychiatry until within recent years the idea of the necessity to provide a broader range of possible interventions gained importance. The first publication reporting data on the use of such measures in a hospital stems from 1991 (29). Beginning from 1997, two voluntary working groups of German hospitals were founded in the Southern and the Northern part of Germany with the aim to analyze and reduce the use of mechanical restraint and other types of coercion and violence (27, 30–32). Since about 2000, after introducing common definitions, first data collections and comparisons between hospitals were made, so-called “benchmarking” in quality circles (33). The most comprehensive data set published so far originates from 10 psychiatric hospitals in the year of 2004 covering 36,690 admissions, another from the other working group reports data from 6 psychiatric hospitals from the same year (2004) covering 10,352 admissions (27). Table 4 presents data as reported in those two studies. All hospitals in these studies used mechanical restraint, only a minority seclusion in addition, the latter to a very different extent. The published data do not provide separate data for seclusion and restraint. Table 2 indicates that differences in the use of seclusion and restraint were considerable between the two studies, and even among the single hospitals of both studies differences were considerable, which is a well-known fact from all countries where data have been published (34, 35).

**Table 4:** **Use of freedom-restrictive coercive interventions (seclusion or mechanical restraint) in German psychiatric hospitals according to ICD-10 first diagnoses**.

Diagnosis	Percentage of admissions exposed to coercive measures (mean) (%)		Cumulative duration of coercive measures per affected case and admission (mean) (h)	
	Steinert et al. (27)	Ketelsen et al. (32)	Steinert et al. (27)	Ketelsen et al. (32)
F0 organic disorders	28.0		96.9	61.4
F1 addictive disorders	4.9		23.9	3.8
F2 schizophrenic disorders	16.1		36.0	15.5
F3 affective disorders	3.4		32.8	6.1
F4 neurotic, anxiety, and somatoform disorders	2.5		22.7	8.8
Personality disorders	9.4		22.3	11.9
All	9.5	3.0	50.6	16.6

Further comprehensive data have not been published since then. Smaller data sets and unpublished results from the participating hospitals indicate that the percentage of admissions exposed to coercive measures and the mean duration of a coercive measure have slightly decreased since then (36).

A survey of the use of coercive interventions in psychiatric hospitals in Germany in 2012 (24) revealed that all hospitals used mechanical restraint. Mechanical restraint without continuous 1:1 supervision still occurred in 37.1% of psychiatric hospitals, in 25% of psychiatric departments at general hospitals and no more at university hospitals. The way how supervision was realized in the hospitals was different: 72% placed a person besides the patient’s bed, 51% supervised through a glass panel, 16% by video, 34% supervised from a distance of no more than a few meters, but without eye contact, and 34% used visits all 1–30 min (some more than one way, therefore over 100%).

### The Netherlands

Whilst seclusion is the measure of first choice, mechanical restraint is seldom used in adult psychiatric care. It is primarily used in old age psychiatry for people with dementia (37). Table 5 shows findings on the use of seclusion, mechanical restraint, and enforced medication over several diagnostic groups as gathered in 2011 (23), displaying the same outcomes as in Table 4 for the German data. These data show that the use of seclusion is higher than in Germany, while the use of mechanical restraint is lower.

**Table 5:** **Use of coercive interventions (seclusion, mechanical restraint, or involuntary medication) in Dutch psychiatric hospitals according to ICD-10 first diagnoses in 2011**.

Diagnosis	No measure (%)	Percentage of admissions exposed to coercive measures (*N* = 38,004) (%)			Cumulative duration of coercive measures per affected case and admission (mean/median)			
		Seclusion (*N* = 4,725)	Restraint (*N* = 379)	Involuntary medication (*N* = 1,128)	Seclusion		Restraint	
					Mean	Median	Mean	Median
F0 organic disorders	88.7	1.5	2.5	1.5	208	28	385	103
F1 addictive disorders	86.5	12.6	1.3	2.3	124	23	404	178
F2 schizophrenic disorders	82.4	17.4	0.6	4.9	165	33	409	7.2
F3 affective disorders	90.5	9.0	0.8	2.1	104	29	215	49
F4 neurotic, anxiety, and somatoform disorders	93.2	6.5	0.5	0.9	166	21	144	4.5
F6 personality disorders	88.6	11.0	0.6	2.0	180	28	0	0
All	88.5	10.9	0.9	2.6	190	32	332	35

## Other Coercive Interventions

### Germany

So-called net-beds or cage-beds, which still are in use in Austria and some other European countries (38) have been in use in Germany until the early 1980s in some places. Since then, such measures are no more in use anywhere to our knowledge. The same applies for other devices such as coercion jackets. However, in old age psychiatry a wide variety of measures is used to protect people with dementia from falls. By definition, all of these measures are subsumed under “mechanical restraint” and comprised in the data of Table 2.

In 2007, a group of German psychiatrists and nurses visited a hospital in the UK to study the practice of physical restraint without mechanical devices. Since then, a working group of nurses developed a new manual-based technique called four-step-program. The technique comprises holding techniques without pain-inducing elements accompanied by continuous verbal de-escalation and offers to the patient to cooperate (39). This approach has gained much interest and has been introduced in several hospitals since then. However, at the time there is no sound study available demonstrating the claimed effects on reduction of time in restraint, acceptance by patients and safety.

“Time out” (order to the patient to stay in his/her own room for a defined time) is mostly used in child and adolescence psychiatry, in adult psychiatry in 13% of the hospitals (24).

### The Netherlands

In the care for people with dementia, net-beds are considered as a better alternative for mechanical restraint. However, the use of “Domotica” (40), which comprises a number of electronic devices, is gaining interest. Such devices have been designed to register movements, but also to measure arousal by means of skin conductance. In several ways, these devices allow monitoring and signaling of out of the order behavior in several groups of patients, both the elderly and patients with a mental disability.

One in one support is considered as a preferable alternative to coercive measures. Also, time out and room programs are viewed as alternatives. Documentation of these measures proved to be less reliable than of seclusion or restraint, primarily because nurses consider these measures as “care as usual” rather than as containment or coercive measures (41).

## Training/Prevention

### Germany

About 20 years ago, de-escalation training for psychiatric hospitals was essentially unknown in Germany. This has continuously been changing since then. After about the year of 2000, de-escalation trainings have been introduced from the Netherlands and the U.S. and became increasingly popular and widespread. Today, private and hospital-based organizations as well offer different kinds of de-escalation techniques and trainings for different patient populations. The training of such techniques for all professionals with patient contact is strongly encouraged by the current German guidelines (42). In the survey among psychiatric hospitals in 2012 (24), 97% of the responding medical directors indicated that some kind of de-escalation training was conducted at their hospital. In 75%, this training followed a plan and half of the respondents indicated that more than 50% of professionals in their hospital had received training at least once a year. However, it is well known from anecdotal evidence that doctors, unlike nurses, are sometimes unwilling to participate in those trainings and it is difficult to ensure that all doctors have received training. Systematic risk assessment techniques generally play a minor role both in training and in clinical practice, different from the Netherlands and, e.g., the UK. Evaluations of all described approaches are scarce or missing.

### The Netherlands

Awareness concerning dangerousness of psychiatric patients at closed wards arised from halfway the 90s (43). Several studies at closed wards emphasized the need for identifying dangers in the interaction between patients and staff within the context of these wards (44, 45). In general, three ways to deal with aggression were developed. The first is aimed at dealing with physically containing the aggressive patient (46), the second primarily with the interaction between the patient and staff (47), while more recently developed training is aimed at dealing with several roles in containing conflict (48). From 2005 onward risk assessment became increasingly important in the training of nurses and mental health professionals in dealing with containing aggression, especially after the nation-wide program to reduce seclusion use was encouraged by the Dutch Government. Since then, several de-escalation training methods have been used together with other measures to reduce seclusion. Only few of these preventive methods have been studied. An exception is the use of daily risk assessment instruments by nurses. Two cluster randomized studies showed that risk assessment reduced the number of aggressive incidents (49, 50) as well as the duration of seclusion (50). Only few hospitals, however, use these methods. A second exception is a cluster randomized trial on the preferred use of enforced medication. Even though the study was flawed by a number of study protocol violations, a 75% reduction of seclusion occurred in the experimental ward.

An evaluation of initiatives within the nation-wide program showed that 92% of Dutch mental health care participated, while all of the participating hospitals provided some way of aggression containment training. From 2011 onward aggression training is obligatory and participation is subject to audits of the Dutch health inspectorate. At least once in 2 years most mental health professionals participate in some kind of training. However, participation of nurses in the program as well as in these trainings is by far higher than of doctors, psychologists, or psychiatrists

## Clinical Guidelines

### Germany

The first guideline on the use of coercive measures, an internal guideline framed by doctors and nurses of our (T.S.) psychiatric hospital, was published in 1998 (51). A national guideline on therapeutic measures for aggressive behavior in psychiatry and psychotherapy, which covers indications for the use of coercive interventions and aspects of human dignity in their realization was published in 2010 (42). The survey among psychiatric hospitals in 2012 mentioned above revealed that all but one of the responding hospitals used an internal guideline or a general guideline such as the German Psychiatric Association’s (DGPPN) guideline (24). Thus a reference to guidelines is the common standard nowadays. However, it is unknown how thoroughly these guidelines are implemented and how much impact they have on the routine clinical practice. Only very little obligatory or supervised common standards for psychiatric hospitals exist except for a legal framework regarding staffing levels in all professional groups.

### The Netherlands

The current clinical guideline was compiled in 2005, which is before the nation-wide effort to reduce seclusion. A new guideline is currently under way. More recently, in line with the English Psychiatric Intensive Care Units (PICU’s) a number of hospitals are developing intensive care as a specialization of Mental health care. Development of intensive care units not only aims at new building environments (28), but also at an increased professionalization of the care provided (52). In 19 psychiatric hospitals, a system of quality audits was set up to investigate the care provided. In these audits, a care quality checklist is discussed by two independent auditors with team nurses and management. Risk assessment, training in dealing with aggression, participation of ex-patients as “experienced workers,” and the use of several environmental alternatives within the ward such as comfort rooms, chill rooms, and rooming in for family members are some of the ways how acute wards can improve the quality of care. The development of intensive care is supported especially by the Dutch Health inspectorate.

## Future and Ongoing Developments

### Germany

The awareness of the ethical and legal problems in the use of any kind of coercive interventions has considerably been increasing during the past years, due to the changes of legislation induced by the constitutional court, continuing criticism by patients’ organizations, criticism by the German Institute for Human Rights, and others and due to public debates on justification of long lasting detention in forensic psychiatry in a special case. This increased awareness is reflected in recent publications in German journals, by an increased importance of the issue in education and training and by changes in legislation. The willingness to reduce the use of coercion and to replace the use of mechanical restraint by softer techniques such as de-escalation and holding is widely present, but to some extent decelerated by concerns of future budget restrictions by the introduction of a new reimbursement system for psychiatric hospitals.

The wide use of electronic charts has considerably improved the possibilities to record all kinds of coercive measures in detail and to perform hospital comparisons. First German federal states will introduce a legal obligation to register coercive measures and to collect them at a central institution in 2014.

Further changes in legislation are also expected, which refers particularly to forensic psychiatry. A reform of the admission criteria, which are intended to be phrased more restrictively, is intended. Currently no details are known, however.

### The Netherlands

In Dutch mental health care, three changes are simultaneously under way. First, the Government together with health insurance offices has been initiating a policy to reduce the number of psychiatric hospital beds by 30% within the next 5 years. This policy was endorsed in 2011, became effective in 2012 and has lead to closure of more than 10% of psychiatric hospital beds over the last 2 years (53). This policy is primarily focused on decreasing the number of long stay beds in favor of the number of acute beds. Also, hospital as well as health insurance policy aims to further decrease the length of stay at acute psychiatric wards.

The second change encompasses the closure of a large number of forensic beds. This closure is not only due to Governmental policy, but also an effect of advice given by an increasing number of lawyers of mentally ill offenders to refuse collaboration with psychiatric observation. Mostly, this observation is not in the interest of the offender as it usually leads to longer time in detainment.

The third change is a pending change in the Law on involuntary admission. In 2015, or at the latest 2016 the current law is to be replaced by two laws regulating involuntary admission as well as involuntary treatment. The first new law will regulate involuntary treatment of psychiatric patients, inside as well as outside of the psychiatric hospital. Under this law, involuntary treatment will be possible under a number of strict conditions. These are related to being a danger for self or a danger for others. The second new law will regulate the involuntary care for patients with a mental disability or a cognitive disorder who are admitted to other than psychiatric services. Both laws aim at treatment rather than at admission. We expect that these laws will have a substantial impact on the distribution of the current figures on coercive measures. While currently seclusion is the measure of first choice and the most used, we expect that this will change when the new law will allow involuntary treatment to a far larger extent than the current law does.

## Discussion

We tried to give a comprehensive overview on the role of coercion in mental health care in Germany and the Netherlands, in terms of clinical practice, policies, ethical views, and the expected future. Mental health care in these neighboring countries features many similarities and interesting differences as well. Both countries have a comparable per capita income and spend comparable percentages of their gross domestic product for health care and mental health care. In both countries, ethical questions around topics of mental health have been repetitively issues of ongoing public debate. However, the historical background is different. In Germany, psychiatry is still (or at least its exponents feel) burdened by the grim heritage of Nazi psychiatry, when psychiatrists and representatives of the states abused the so far well-doing health care system to record, sterilize, and later kill 10,000 of patients. Against this background, for example the German attitude to euthanasia is very different to the Netherlands, where a relatively liberal practice has been legalized in recent decades. In Germany, instead, the code of medical ethics explicitly forbids physicians even any assistance in suicide, even if it may not be unlawful. Similarly, whatever psychiatrists and judges do against a patient’s will, in Germany always is under latent suspicion of Nazi psychiatry. Nonetheless, the legal framework for involuntary admission and detention of mentally ill people is rather similar in Germany and the Netherlands. Also the rate of involuntary admissions per 100,000 inhabitants is somewhat lower in the Netherlands, but not to a striking extent, and the percentage (quota) of involuntary admissions to psychiatric hospitals is nearly identical. However, the rise of the quota of involuntary admissions within the past 10 years, which has been found in the Netherlands could not be confirmed for Germany. The reasons are unknown.

In some aspects, the practice of the countries has fertilized each other. De-escalation and aggression-management trainings have been introduced in Germany by commercial trainers from the Netherlands about 15 years ago. By now such trainings are recommended by guidelines and implemented in routine practice in most psychiatric hospitals (24). On the other hand, the system and the outcome measures developed to compare the use of coercive measures among different hospitals in Germany have been adopted in the Netherlands. But the Netherlands then succeeded earlier than Germany to establish a country-wide database for the use of coercive measures, which there is viewed as a task for the future, hampered by the existence of 16 different mental health laws in the respective federal states.

Most striking, however, is the diverging development of attitudes toward the use of different coercive interventions. For a long time, the use of coercive medication was viewed as most restrictive intervention in the Netherlands, being an intrusion into the body. Accordingly, legal requirements were high and, in practice, remained confined to emergency situation, since psychiatrists themselves held the same attitude. However, becoming aware that reported aggressive incidents in psychiatric hospitals as well as number and duration of seclusions were higher than in any other European country (22), the assumption that this was the consequence of the extensive ban of medication got increasingly accepted and opinions begun to change. So within recent years there has been a still ongoing change in clinical practice in the Netherlands, moving from the sole use of seclusion to early intervention by drugs, if necessary by use of coercion, and including not only in-patients but also out-patients in future, based on revised legal framework. This change of clinical practice has been encouraged by data from other countries such as Germany and recent studies in the Netherlands, which could demonstrate that a preferred use of medication can substantially reduce the use of seclusion (54) and that involuntary medication causes less subjective distress than seclusion or restraint (41).

Germany, however, seems to be on a way just in the direction where the Netherlands came from. Until 2011, the use of involuntary medication was widely accepted, possible in involuntarily committed patients and viewed as therapy, not as a mode of restraint (a German equivalent of “chemical restraint” is completely uncommon in clinical language). Only for patients committed by Guardianship law a separate decision by a judge was required. Since the decisions of the Constitutional Court in 2011, there has been a considerable change in opinions held about coercive medication, but just in the other direction than in the Netherlands. Though laws have been revised since then and coercive medication is possible again under the strict requirements defined by the Constitutional Court, psychiatrists have recognized that it has been possible in most cases to convince patients to accept treatment without coercion and they rarely apply at courts for the respective intricated procedures. Attitudes of physicians, patients’ representatives, and the general public toward the use of coercive medication seem to have become more critical. The change of attitude is best characterized by the statement by the Ethics Committee at the Federal Chamber of Physicians published in 2013 (55), which explains that the use of coercive medication is the most invasive measure and that in case of danger to others mechanical measures such as detention would be less restrictive and consequently preferable, leaving open the interpretation that even restraint should be preferred to medication.

Importantly, evidence does not seem to play a role in most of discussions on the issue. Studies showed that patients do not necessarily prefer one coercive practice above the other; in several studies it was found that in case of a need for a coercive measure almost half of patients prefer medication, and the other half prefer seclusion (56). Ideally, patients should be able to state their preference in a form of advance statement, to match patients’ wishes to the practice used.

One other large difference in coercive practices is the use of outpatient commitment and involuntary treatment in the Netherlands as opposed to Germany. Even the new Dutch law that will be in practice the coming years, heavily invests in outpatient involuntary treatment, thereby hoping to reduce involuntary admissions. Scientific evidence, however, points in another direction, since all three randomized clinical trials studying outpatient commitment found that outpatient commitment did not lead to a reduction of the number of (in)voluntary admissions (57–59).

Further differences between the countries strike with respect to the culture of setting standards and evaluations. In the Netherlands with the Dutch health inspectorate there is a governmental authority having the power to enforce changes in practice and the power to phrase and control obligatory standards such as for intensive care units. The awareness of the need to evaluate actions taken and to base political decisions on available evidence is not really widespread but is at least increasing. In Germany, in contrast, the federal government is not responsible for mental health care, which is under regulation of 16 different states instead. Hospitals are led by different public, private, and confessional providers, and the German Society of Psychiatry and Psychotherapy (DGPPN) basically is a club of psychiatrists with no political authority. Therefore, there is no control whether guidelines are followed, quality standards are based mostly on agreement and evaluation of measures has been scarce.

For the future, we hope that both countries will benefit from the observation of the developments in the respective other country and include evidence from scientific studies into legislation and political decision making, realizing a reasonable, evidence-based practice committed to therapeutic goals, and human dignity in a modern civil society.

## Conflict of Interest Statement

The authors declare that the research was conducted in the absence of any commercial or financial relationships that could be construed as a potential conflict of interest.
